# Effects of Surgical Treatment Guided by the Three-Column Classification Method on Knee Joint Function and Postoperative Complications in Patients with Tibial Plateau Fractures

This article has been retracted.

**DOI:** 10.1155/2022/5935102

**Published:** 2022-05-09

**Authors:** Jiayi Guo, Yuan Liu, Yiran Feng, Lin Zhang, Feng Li, Yunfei Zhang, Zhenya Wang, Yongbing Wen, Yanxing Guo

**Affiliations:** ^1^Luoyang Orthopedic Hospital of Henan Province (Orthopedic Hospital of Henan Province), Luoyang 471002, Henan, China; ^2^New Zealand College of Chinese Medicine, Auckland, New Zealand

## Abstract

Many patients with tibial plateau fractures present with various degrees of soft tissue contusion and severely damaged articular surface, ligament, and vascular nerves, and thus how to treat this kind of patient has become one of the great difficulties in clinical practice. Therefore, we aim to investigate the effects of surgical treatment guided by the three-column classification method on knee joint function and postoperative complications in patients with tibial plateau fractures. A total of 120 patients with three-column tibial plateau fractures admitted to our hospital from January 2018 to January 2019 were selected and divided into group A (*n* = 60) and group B (*n* = 60). Among them, the group A patients were treated with an anterior lateral approach in floating positions combined with reduction plate internal fixation with an L-shaped approach in the posteromedial joint, while the patients in group B received reduction plate internal fixation with a knee midline incision in supine positions. After that, the perioperative indexes, knee function scores, the MOS item short-from health survey (SF-36) scores, complication rate (CR), and overall treatment efficacy of the patients were compared between the two groups. The perioperative indexes in group A were significantly better than those in group B (*P* < 0.001); the knee function scores and SF-36 scores in group A were significantly higher than those in group B (*P* < 0.001); the CR in group A was significantly lower than that in group B (*P* < 0.001); the treatment efficacy in group A was significantly better than that in group B (*P* < 0.05). The three-column classification method, with highly instructive significance in tibial plateau fracture surgery, can improve treatment efficacy and reduce the incidence of complications, which is worthy of application and promotion in clinical practice.

## 1. Introduction

Tibial plateau fractures commonly refer to intraarticular fractures mostly caused by high-energy injuries or even slight strike in the elderly, and the minority of patients suffering from such fractures present with soft tissue and nerve injuries, which have still not been treated properly and completely until now and can lead to poor prognosis in patients. Therefore, this condition requires a prompt interventional surgery for the sake of protecting patients' knee joint function, which should be conducted with stringent specification as the differences in various approaches have a decisive effect on treatment efficacy. Also, the traditional treatment guided by the Schatzker classification has some drawbacks in terms of precision, especially in describing posterior tibial plateau fractures in patients.

Studies conducted in recent years have shown that the traditional theory of fracture classification has been unable to meet clinical needs. For example, the theoretical basis of Schatzker classification is two-dimensional images, characterized by superposition, thus hardly fully demonstrating the spatial relationship of the tibial plateau and then leading to some errors. However, the theory of three-column classification, in which the tibial nodes are classified as point A, internal angle tibia point B, anterior fibular head point C, and midpoint of tibial spine point O and the connecting line among these 4 points divides tibial plateau into 3 parts, proposed by the scholar Congfeng Luo, enables orthopedists to enrich their perceptions of disparate fracture types and then enhance the scientificity in the selection of surgical approaches, comprehensively optimizing the therapeutic effects of the surgical treatment for tibial plateau fractures [1–3]. In addition, recent studies have revealed that the clinical guiding significance of the three-column classification method is better than that of routine classification.

Therefore, we proposed to explore the effects of surgical treatment guided by the three-column classification method on knee joint function and postoperative complications in patients with tibial plateau fractures. We have chosen 120 patients with tibial plateau fractures admitted to our hospital from January 2018 to January 2019 as the study subjects. The dataset was divided into group A (*n* = 60) and group B (*n* = 60). Also, we have analyzed the results thoroughly.

## 2. Materials and Methods

### 2.1. General Information

A total of 120 patients with three-column tibial plateau fractures admitted to our hospital from January 2018 to January 2019 were selected and divided into group A (*n* = 60) and group B (*n* = 60). There were no significant differences in the general information of the patients between the two groups (*P* > 0.05), with research significance, as shown in Table 1.

### 2.2. Inclusion Criteria

(1) Patients and their family members were informed of the purpose and process of the study and signed the informed consent. (2) Patients were diagnosed with tibial plateau fractures by the imageological examination and met the criteria for three-column classification. (3) This study was approved by the Hospital Ethics Committee.

### 2.3. Exclusion Criteria

(1) Patients had mental disorders or could not communicate with others. (2) Patients suffered from other severe organic diseases.

### 2.4. Methods

#### 2.4.1. Treatment in Group A

After receiving epidural anesthesia, the patients took floating positions for surgery. During surgery, patients' articular capsules were incised to observe the conditions of meniscus and cruciate ligaments, and subsequently the lateral tibial plateau was visualized in the field of view. At the same time, the patients' collapsed articular surface was raised and fixed with metal pins (manufacturer: Shanghai Simz Jinhuan Medical Products Co. Ltd.; State Food and Drug Administration Certified No. (2014) 3461568).

After that, patients' positions moved forward. An L-shaped approach incision on patients' posterior knee joint was performed, and then the medial head of gastrocnemius was pulled apart to make the posterior tibial plateau visible. The collapses and fractures of patients were reduced and fixed with metal bone needles. The reduction was observed with an X-ray machine (Manufacturer: Xi'an Land Com Digital Medical Science and Technology Co., Ltd.; Shan Xi Food and Drug Certified No. (2009) 2300118). After the reduction, the posterior tibial plateau was fixed with a T-type plate.

For the patients requiring visualization of the medial column, the incision was stripped forward, and after reduction and fixation, the tissues were sutured. For the patients with severer bone defects, allogeneic bones were used and fixed with a proximal lateral tibial anatomical plate, followed by sutures and cross fixation with absorbable wires.

Patients' surgical wounds were irrigated and sutured, with the aid of a negative pressure drainage tube.

#### 2.4.2. Treatment in Group B

The anesthesia methods adopted in group B were the same as those in group A. Patients' anterior median incision was taken, and their joint capsules were incised according to the fracture site. For the patients with the collapse of the articular surface, the articular surface was reduced and fixed by metal pins then.

The flap was detached from the outside of the incision so that the fracture end of the lateral tibial plateau was presented in the field of view. Subsequently, the joint capsules were incised to observe the actual conditions, and the meniscus was raised to make lateral tibial plateau visible. Then, the percutaneous reduction by leverage was performed and the metal pins were used to reduce the lateral tibial plateau. The X-ray machine was used to observe the reduction conditions, and the fixation with a plate was conducted for patients. The performance of the suture and the placement of negative pressure tubes were both same as those in group A.

#### 2.4.3. Observation Indexes

(1) Perioperative indexes included the operation time, intraoperative blood loss, postoperative drainage volume, postoperative ambulation time, and postoperative weight-bearing time. (2) Knee joint function score: the Rasmussen scale was used to evaluate the knee joint function of patients, with the score ranging from 0 to 30 points, and higher scores indicated better knee joint function; the ROM was adopted to judge the joint mobility of patients, and higher scores indicated better joint mobility [4–7]. (3) SF-36 score: the SF-36 scores at 3, 6, and 9 months after surgery were compared, and higher scores represented healthier conditions [8–11]. (4) CR: the occurrence of complications such as delayed healing, deep infection, superficial infection, and lower extremity deep venous thrombosis was recorded. (5) Overall efficacy: patients' treatment efficacy was evaluated by the American Hospital for Special Surgery (HSS) scale, in which scores of 90 and above were considered excellent, those between 80 and 89 were considered good, and those in the range of 79 and below were considered poor [12–15].

#### 2.4.4. Statistical Treatment

The selected data processing software for this study was SPSS20.0, and the software selected to draw the pictures of the data was GraphPad Prism 7 (GraphPad Software, San Diego, USA). Measurement data were tested by *t*-test and enumeration data were tested by X^2^ test. The differences had statistical significance when *P* < 0.05.

## 3. Results

### 3.1. Comparison of Perioperative Indexes between the Two Groups

The perioperative indexes in group A were significantly better than those in group B (*P* < 0.001), as shown in Table 2.

### 3.2. Comparison of Knee Joint Function Scores between the Two Groups

The knee joint function scores in group A were significantly higher than those in group B (*P* < 0.001), as shown in Figures 1 and 2.  Figure 1 shows that the Rasmussen scores were (27.0 ± 2.5) points in group A and (21.0 ± 2.1) points in group B.  Figure 2 shows that the ROM was (27.0 ± 2.5) points in group A and (21.0 ± 2.1) points in group B.

### 3.3. Comparison of SF-36 Scores between the Two Groups

The postoperative SF-36 scores in group A were significantly higher than those in group B (*P* < 0.001), as detailed in Figure 3. From Figure 3, we can see that at *T*_0_, the SF-36 scores were (52.1 ± 5.1) points in group A and (45.2 ± 5.2) points in group B. Also, at T1, the SF-36 scores were (76.2 ± 6.0) points in group A and (68.0 ± 3.2) points in group B. At *T*_2_, the SF-36 scores were (90.2 ± 1.2) points in group A and (82.3 ± 3.2) points in group B.

### 3.4. Comparison of CR between the Two Groups

The CR in group A was significantly lower than that in group B (*t* = 62.484, *P* < 0.001), as shown in Figure 4. From Figure 4, we can conclude that delayed healing occurred in 0 patients in group A and 2 patients in group B, deep infection occurred in 1 patient in group A and 2 patients in group B, superficial infection occurred in 2 patients in group A and 4 patients in group B, and DVT occurred in 2 patients in group A and 4 patients in group B. There were 55 patients with no complications in group A and 48 patients with no complications in group B.

### 3.5. Comparison of Overall Efficacy between the Two Groups

The treatment efficacy in group A was significantly better than that in group B (*P* < 0.05), as shown in Table 3.

## 4. Discussion

In general, conservative treatment cannot exert obvious therapeutic effects, while surgery is carried out more commonly under the premise of classified fractures that are of great significance to determining the selection of appropriate surgical approaches [4, 16–19]. Therefore, a new means of fracture classification resorted by the latest three-dimensional imaging technology is imperative. The three-column classification theory based on the three-dimensional imaging results of CT scanning proposed by the scholar Congfeng Luo, as mentioned above, divides the tibial plateau into three parts, which enables medical staff to understand the fracture types of the tibial plateau in depth and provide more scientific references for the preparation of surgical protocols [20–23].

In this study, the perioperative indexes in group A were significantly better than those in group B, and the knee joint function scores and SF-36 scores in group A were significantly higher than those in group B (*P* < 0.001), indicating that based on the three-column classification theory, an anterior lateral approach in floating positions combined with reduction plate internal fixation with an L-shaped approach in the posteromedial joint can improve surgical efficiency. In addition to the improved therapeutic effects, guided by this theory, the problems of fewer anterior tibial plateau muscles and thinner blood flow in patients were solved, and the surgery was carried out smoothly, with a higher success rate of fracture reduction, revealing that the procedure guided by the three-column classification method can improve patients' prognosis and promote their desirable recovery.

Furthermore, patients may encounter the problem of unstable fracture fixation during treatment, and in severe cases, complications such as skin necrosis may occur, negatively affecting surgery effects and postoperative rehabilitation progress, so reducing the incidence of complications is also an important aim of surgical implementation. Our study results showed that the CR in group A was significantly lower than that in group B (*P* < 0.001), and the overall efficacy in group A was better than that in group B (*P* < 0.05), which are consistent with the conclusions drawn from the scholar Yusof, who adopted the three-column classification method and treatment plans (same as those in our study) for the two groups in his study and found that the patients in the experimental group had the CR of 9.0 % (9/100), which was significantly lower than that in the control group [24], confirming that under the guidance of routine fracture classification theory, patients are more likely to suffer from surgical complications, greatly reducing therapeutic effects. The surgical protocol based on the theory of three-column classification can fully expose the lateral column through a posteromedial approach, which makes the reduction more targeted and easier; an L-shape incision can reduce the incidence of failing reduction of several poor bone blocks, greatly decreasing CR and improving overall outcomes.

## 5. Conclusion

In conclusion, our study results showed that under the guidance of routine fracture classification theory, patients are more likely to suffer from surgical complications, greatly reducing therapeutic effects. Also, the surgeries guided by the three-column classification method for the treatment of tibial plateau fractures can optimize surgical indexes, improve the recovery of knee joints, and reduce the incidence of complications in patients, which is worthy of application and promotion in clinical practice. However, there are still some limitations in our study. For example, the dataset was still limited. Therefore, we need to collect more patients' information to conduct our experiments.

## Figures and Tables

**Figure 1:** Comparison of knee joint function scores between the two groups ($\bar{x}$ ± *s*, points). Note: the abscissa represented groups A and B, while the ordinate represented Rasmussen score (points). ^*∗*^ indicated *P* < 0.001.

**Figure 2:** Comparison of ROM between the two groups ($\bar{x}$ ± *s*, °). Note: the abscissa represented groups A and B, while the ordinate represented ROM (°). ^*∗*^ indicated *P* < 0.001.

**Figure 3:** Comparison of SF-36 scores between the two groups ($\bar{x}$ ± *s*, points). Note: the abscissa represented 3 months (T0), 6 months (T1), and 9 months (T2) after surgery, while the ordinate represented SF-36 score (points). ^*∗*^ indicated *P* < 0.001.

**Figure 4:** Comparison of CR between the two groups (*n* (%)). Note: the black area represented delayed healing, the dark gray area represented deep infection, the grid area represented superficial infection, the white area represented DVT, and the light gray area represented no complications.

**Table 1:** Comparison of general information between the two groups.

Group	Cases	Male to female ratio	Average age (years old)	Schatzker		Time from getting fractures to the beginning of surgery (d)
				V	VI	
Group A	60	33/27	39.5 ± 5.1	35	25	9.0 ± 1.2
Group B	60	32/28	39.1 ± 5.1	34	26	9.1 ± 1.3
X^2^/*t*		0.034	0.430		0.034	0.438
P		0.855	0.668		0.853	0.662

**Table 2:** Comparison of perioperative indexes between the two groups ($\bar{x}$ ± *s*).

Group	Operation time (min)	Intraoperative blood loss (ml)	Postoperative drainage volume (ml)	Postoperative ambulation time (d)	Postoperative weight-bearing time (d)
Group A	130.2 ± 6.5	201.2 ± 12.0	52.3 ± 10.1	4.1 ± 0.8	40.0 ± 10.2
Group B	145.2 ± 5.4	218.3 ± 12.5	62.3 ± 10.5	7.2 ± 0.9	49.3 ± 11.0
*t*	13.750	7.644	5.317	19.941	4.802
P	0.000	0.000	0.000	0.000	0.000

**Table 3:** Comparison of overall efficacy between the two groups (*n* (%)).

Group	Excellent	Good	Poor	Excellent and good
Group A	28 (46.7)	30 (50.0)	2 (3.3)	58 (96.7)
Group B	18 (30.0)	32 (53.3)	10 (16.7)	50 (83.3)
X^2^	3.525	0.134	5.926	5.926
P	0.060	0.715	0.015	0.015

## Data Availability

The datasets used and/or analyzed during the current study are available from the corresponding author on reasonable request.
